The article "Brain MRI Radiomics Analysis of School-Aged Children with Tetralogy of Fallot" was published in 2021. Journal: Comput Math Methods Med.

# Brain MRI Radiomics Analysis of School-Aged Children with Tetralogy of Fallot

**DOI:** 10.1155/2021/2380346

**Published:** 2021-10-29

**Authors:** Yiwei Pu, Songmei Li, Siyu Ma, Yuanli Hu, Qinghui Hu, Yuting Liu, Mengting Wu, Jia An, Ming Yang, Xuming Mo

**Affiliations:** ^1^Department of Cardiothoracic Surgery, Children's Hospital of Nanjing Medical University, Nanjing, China; ^2^Department of Cardiac Surgery, The Second Affiliated Hospital of Harbin Medical University, Harbin 150086, China; ^3^Department of Radiology, Children's Hospital of Nanjing Medical University, Nanjing, China

## Abstract

**Introduction:**

Radiomics could be potential imaging biomarkers by capturing and analyzing the features. Children and adolescents with CHD have worse neurodevelopmental and functional outcomes compared with their peers. Early diagnosis and intervention are the necessity to improve neurological outcomes in CHD patients.

**Methods:**

School-aged TOF patients and their healthy peers were recruited for MRI and neurodevelopmental assessment. LASSO regression was used for dimension reduction. ROC curve graph showed the performance of the model.

**Results:**

Six related features were finally selected for modeling. The final model AUC was 0.750. The radiomics features can be potential significant predictors for neurodevelopmental diagnoses.

**Conclusion:**

The radiomics on the conventional MRI can help predict the neurodevelopment of school-aged children and provide parents with rehabilitation advice as early as possible.

## 1. Introduction

Radiomics, a rapidly emerging field of medical image, could be potential imaging biomarkers by capturing and analyzing the features, such as shape and heterogeneity [1]. Radiomics features along with demographic, histologic, genomic, and proteomic data can discover and solve lots of clinical problems [2]. Radiomics focuses on phenotypic signatures in neurological and neuropsychiatric disorders [3] and can assist in the diagnosis of neoplastic and nonneoplastic disorders in the brain. The guideline from the European Association of Neuro-Oncology (EANO) has added radiogenomics as a diagnosis and treatment of adult glioma [4]. Besides, a recent study showed that the patients with attention deficit hyperactivity disorder (ADHD) can be separated from healthy control subjects by cerebral radiomics-based classification models [5]. A study on preterm infants also suggested that texture analysis of deep medullary veins (DMVs) on susceptibility-weighted imaging (SWI) can be potentially used for identifying ischemic injury [6]. However, few studies addressed the cerebral radiomics changes in congenital heart disease (CHD) children whose neurodevelopment was paid increasing attention recently [7, 8].

Children and adolescents with CHD have worse neurodevelopmental and functional outcomes compared with their peers, although the development of the patients' life support and operative techniques contributed to higher levels of overall survival [9]. In particular, children with complex CHD were vulnerable to neurological disorders [10]. Except the cerebral developmental delayed in many infants with CHD, brain injuries such as decreased cerebral blood flow (ischemia) and included (punctate) white matter injury, periventricular leukomalacia, and stroke are always reported [11]. Meanwhile, those CHD patients often have difficulties with social cognition and executive functioning while their neurodevelopmental scales were within the normal ranges in the early period [10, 12, 13]. Therefore, early diagnosis and intervention are the necessity to improve neurological outcomes in CHD patients.

Since the past century, researchers have tried to find difference between the CHD patients and healthy peer group by MRI [14, 15]. At first, brain injury was confirmed in patients after surgery [16]. Then, studies reported structural brain abnormalities appearing before surgical intervention [17, 18]. Not only that, more studies centered on the predictive skill of MRI for neurodevelopmental outcomes or the correlation effects of them were published during the recent last decade [19–26].

However, it is important to realize that the problem is that these results rely on specific imaging techniques. It is worth thinking about how to predict the neurodevelopment and function of school-aged children and how to provide parents with rehabilitation advice as early as possible.

## 2. Materials and Methods

### 2.1. Enrolled Patients

This study was approved by the Research Ethic Committee of Children's Hospital of Nanjing Medical University and performed in accordance with the code of ethics of the Declaration of Helsinki for experiments involving humans. All data were anonymous during the processing. From November 2015 to June 2016, we recruited 9 school-aged TOF patients from the Children's Hospital of Nanjing Medical University who had undergone corrected surgery before. Nine healthy controls were matched to TOF patients in terms of age, gender, and education. All participants are not diagnosed as hereditary syndromes or any diseases of the central nervous system, and informed consent was acquired from the children and the children's legal guardians. None of them had contraindications to MRI.

### 2.2. MRI Data Acquisition and Preprocessing

MRI data were acquired from all participants using a 1.5 T MRI machine (Siemens Magnetom Avanto, Erlangen, Germany) with a standard 12-channel head coil. T1-weighted MRI data were obtained using the following parameters: TR = 1900 ms, TE = 2.48 ms, TI = 900 ms, image matrix = 256 × 256 × 176, and voxel resolution = 1 × 1 × 1 mm^3^.

The scanning time was 6 min. All participants were prevented from scanner noise by sponge plugs and requested to lie awake quietly with their eyes closed and avoid thinking. During the scans, the subject's head was braced with foam padding to minimize movement artifacts.

The original DICOM data were converted to the format of NIfTI file format by using MRIcron (https://www.nitrc.org/projects/mricron). This modification was accomplished using the following steps [7]: (1) removal of data from the first 10 time points, (2) correction of slice timing, (3) correction of head movements and exclusion of cases that head movement exceeded 1 mm of translation or 1° of rotation about the *x*, *y*, or *z* axis, (4) spatial registration and linear detrending, (5) low-frequency filtering (0.01–0.08 Hz), and (6) half-maximum (FWHM) = 4 × 4 × 4 mm^3^.

### 2.3. Radiomics Feature Extraction and Selection

We selected the region of interest (ROI) in the brain of all patients using 3D slicer (version 4.8.0; http://www.slicer.org). The feature extraction was performed with the open-source Pyradiomics package (http://www.radiomics.io/pyradiomics.html). For T1WI [27], 851 radiomics features (18 first-order features, 14 shape-based features, 75 textural features, and 744 transform-based features) were extracted from each ROI. The least absolute shrinkage and selection operator (LASSO) logistic regression algorithm, with penalty parameter tuning conducted by 10-fold cross-validation, was used to select CHD-related features. The workflow for this procedure is shown in Figure 1.

### 2.4. Neurodevelopmental Outcomes and Clinical Factors' Selection

The neurodevelopmental abilities of children were evaluated by the Wechsler Intelligence Scale for Children–Chinese revised edition (WISC-CR). The WISC-CR, commonly accepted for use in this population [28], is composed of 6 verbal and 6 performance subscales. The full-scale intelligence quotient (FSIQ) is derived from verbal intelligence quotient (VIQ) and performance intelligence quotient (PIQ) calculated by these 12 domains. Clinical variables including birth history were collected from the electronic medical records.

### 2.5. Statistical Analysis

Clinical characteristics of the subjects were described as the mean ± SD. The two-sample *t*-test and the nonparametric Mann–Whitney *U* test (*U*) were considered significant when *p* < 0.05 in the process of dimensionality reduction. The *χ*^2^ test was used to compare the sex distributions between the groups. The LASSO linear regression was performed for the final model. The diagnostic performance of established models was evaluated by receiver operator characteristic (ROC) curves.

These above analyses were performed in SPSS (version 26, https://www.ibm.com/analytics/spss-statistics-software) or R software (version 4.1.0, http://www.r-project.org).

## 3. Results

### 3.1. Characteristics and Neurodevelopmental Outcomes

The demographic characteristics and the intelligence score of the TOF and HC groups are shown in Table 1. No significant difference was observed in age, gender, or years of education. Although the mean FSIQ of these children with TOF was within the range of normal intelligence, it was lower than the mean FSIQ of the HC group and of statistically significant differences.  Table 2 shows the clinical characteristics and neurodevelopment assessment of the TOF patients. Likewise, there was no significant difference observed in age, gender, or years of education.

### 3.2. Radiomics Analysis

Of the 851 extracted features, 393 features (15 first-order features, 8 shape-based features, 28 textural features, and 342 transform-based features) with high reproducibility were selected for subsequent analysis (Figure 2). Six related features shown in Table 3 were finally selected.

### 3.3. Performance and Validation of the Established Model

At first, including all the selected features in a logistic regression model resulted in overfitting. Separate regressions were conducted for each feature. All the six features were shown high confidence for distinguishment by ROC analysis. Correlations were calculated using the Spearman correlation. No significant correlations were observed with wavelet-HHH first-order skewness (Figure 3).

Next, two features with zero coefficients were included to the new logistic regression model. Two models of them were shown overfitting. Two had no statistical significance. The other predicted effects are shown in Figure 4 and Table 4.

Finally, wavelet-HHH first-order skewness and original first-order interquartile range were included to the final model. The AUC value of FSIQ greater than or equal to 100 based on the radiomics was 0.75 (Figure 5).

## 4. Discussion

This was the first using radiomics to investigate the MRI of children with CHD and predict the neurodevelopmental outcome.

MRI was an efficient method to identify brain regions in some cohort of preterm children [29–31]. It is also one of the most efficient tools for clinicians and researchers to evaluate the developing brain [32, 33]. About half of the children with CHD were found to have abnormalities in MRI before surgery [34–37], while most of them have been reported no abnormal neonatal MRI findings [38]. Moreover, mild ischemic lesions shown on MRI in the neonatal periods completely disappeared 4 to 6 months after surgery [16]. However, more and more studies confirm that the adolescents and adults suffer from frequent neurodevelopmental challenges, including cognitive, motor, language, psychosocial, social, and communication impairments [13, 23, 39, 40]. Experts interrogate the association between brain abnormalities and function, such as brain volume [41, 42], hemispheric sulcal patterns [43–45], and white matter microstructure.

It is worth noting that some of the preterm children having no cerebral palsy on normal scans were observed to have poor motor outcomes [46]. For these specific children, a previous study found that a radiomics approach predicts poor psychomotor outcome at a corrected age of 12 months [27], which indicated that radiomics has a significant effect on the predictive value of neurodevelopmental assessment.

Previous studies suggested that some structural brain abnormalities such as the focal and multifocal lesions [23], white matter injury, reduced brain volume, and thinner cortex could be detected by T1WI. With the rapid advances in modern imaging techniques and application, a variety of new image sequences (Flair (fluid attenuated inversion recovery), SWI, DTI (diffusion tensor imaging), fsMRI (fast magnetic resonance imaging), DWI (diffusion-weighted imaging), DKI (diffusion kurtosis imaging), PWI (perfusion imaging), MRS (magnetic resonance spectroscopy), DCE- (dynamic contrast-enhanced-) MR, and BLOD-fMRI (blood oxygenation level-dependent-functional magnetic resonance imaging)) were validly noninvasive diagnostic test for patients with CHD [7, 44]. However, those new image sequences required high costs, high-end equipment, and specific professionals; and neuroimaging was still unable to accurately predict neurodevelopment in children affected by CHD. Deeper analyses on the conventional MRI seemed to be more economical and have wider applicability.

In this study, we chose the radiomics biomarkers from whole-brain MRI due to the lack of a well-recognized mask for children. Contrary to the diagnosis of imaging, the analysis of radiomics is severely affected by masks which automatically delineate ROIs [47, 48]. We trade off the assignment of brain regions to achieve higher concordance within its problem domain. However, delineating the outline of the brain regions has implications for investigating the potential mechanisms of pathogenesis.

Considering the limit cases, we selected the statistically significant radiomics feature between the patients with TOF and the healthy control for dimensionality reduction. The smaller cohort size caused overfitting in the model built by binary logistic regression analysis. Many major features were significantly more relevant if obtained from wavelet-transformed images [49].

As shown in many other studies, patients with TOF were usually tested as low-normal intelligence quotient (IQ). Most of them were not diagnosed as intellectual impairment by neuropsychological testing [43, 50]. This agreed with our results. However, some investigators have previously found that patients with low-normal IQ have higher possibility in progressing to abnormal neurodevelopment [51–53]. Considering these current studies and clinical reality, we preferred 100 rather than 80 as the cut-off of FSIQ. During the selection of features, the data of healthy control was applied for primary screening due to the richness of radiomics features and the small sample sizes compared with the usual ones.

Additional studies are necessary to find more imaging biomarkers and radiomics evidence. In order to translate biomarkers into clinical practice, rigorous technical, biological, and clinical validation is needed [49]. The new guidelines and standards are set by the European Imaging Biomarkers Alliance (EIBALL) and Quantitative Imaging Biomarkers Alliance (QIBA), which standardize the procedure of case inclusion, MRI protocols, feature extraction, and so on [1, 2], although it is established for neuro-oncology, so as in neuroimaging.

This study has a number of limitations. First, the limited number of cases in this study prevents robust confidence from our analysis. Radiomics data are mineable that usually rely on sufficiently large datasets. Considering the uncommon disease entity, the cases are adequate to offer initial screening efforts and the overall modeling. Second, the MRI is used to anticipate future neural development in majority of studies targeting CHD patients. We failed to make regular telephone or mail contact with these participants. In other following studies, we will try to interrogate the prediction of conventional MRI for late neural development. Finally, our models have not yet been externally validated, and thus, the generalizability of the models to other populations remains unknown. Most published studies on radiomics have the same shortcomings [1].

## 5. Conclusion

The radiomics on the conventional MRI can help predict the neurodevelopment of school-aged children and provide parents with rehabilitation advice as early as possible. Moreover, the radiomics signature may work as an independent prognostic factor for diagnoses of brain development-related disorders.

## Figures and Tables

**Figure 1:** Workflow of necessary steps in this study. ROI was delineated on T1WI. Radiomics features including first-order statistics, shape-based features, textural features, and wavelet transforms were extracted. LASSO regression was used for feature selection. The performance of established models was evaluated by ROC curves and Spearman analysis. ROI: region of interest; LASSO: least absolute shrinkage and selection operator; ROC: receiver operator characteristic.

**Figure 2:** Selections of radiomics features. (a) Optimal *λ* value was determined by the LASSO model using 10-fold cross-validation via minimum criteria. The binomial deviance curves were plotted versus log(*λ*). (b) LASSO coefficient profiles of the 6 selected features were presented.

**Figure 3:** The performance of established models was evaluated by ROC curves and Spearman analysis. ROC: receiver operator characteristic.

**Figure 4:** The performance of established models was evaluated by ROC curve. ROC: receiver operator characteristic.

**Figure 5:** Wavelet-HHH first-order skewness and original first-order interquartile range were included to the final model. The performance of established models was evaluated by ROC curve. ROC: receiver operator characteristic.

**Table 1:** Characteristics of the study population.

Variables	TOF (*n* = 9)	HC (*n* = 9)	*p* value
Age (year)	9.55 ± 1.04	9.75 ± 0.65	0.699
Sex (male/female)	5/4	6/3	0.730
Education (year)	2.16 ± 1.22	2.35 ± 0.43	0.438
VIQ	94.00 ± 13.85	122.00 ± 9.14	**0.004**
PIQ	96.00 ± 17.00	104.20 ± 12.76	0.364
FSIQ	94.33 ± 15.09	115.40 ± 10.21	**0.019**

Mean ± SD. TOF: tetralogy of Fallot; HC: healthy children; VIQ: verbal intelligence quotient; PIQ: performance intelligence quotient; FSIQ: full-scale intelligence quotient. Bold values represent that the results have statistical significance.

**Table 2:** Characteristics of the patients.

Variables	FSIQ ≥ 100	FSIQ < 100	*p* value
Age (year)	9.45 ± 1.17	9.67 ± 1.01	0.905
Sex (male/female)	3/2	2/2	1.000
Education (year)	2.28 ± 1.34	2.00 ± 1.24	1.000
VIQ	104.20 ± 8.87	81.25 ± 4.03	**0.016**
PIQ	107.80 ± 7.53	81.25 ± 13.15	**0.016**
Age of surgery (year)	1.97 ± 1.70	1.94 ± 2.25	1.000
Hospital stays (day)	17.00 ± 3.46	19.33 ± 8.62	0.629

Mean ± SD. VIQ: verbal intelligence quotient; PIQ: performance intelligence quotient; FSIQ: full-scale intelligence quotient. Bold values represent that the results have statistical significance.

**Table 3:** List of radiomics features to classify neurodevelopment in TOF and HC groups.

Image type	Feature type	Radiomics feature
Original	First order	Interquartile range
Wavelet-LLH	First order	Kurtosis
Wavelet-LHL	GLSZM	Small area high gray level emphasis
Wavelet-HLH	NGTDM	Complexity
Wavelet-HHL	GLSZM	Small area high gray level emphasis
Wavelet-HHH	First order	Skewness

H: high-pass filter; L: low-pass filter; GLSZM: gray level size zone matrix; NGTDM: neighborhood gray-tone difference matrix.

**Table 4:** Summary of LASSO logistic regression.

	Estimate	Std. error	*z* value	Pr(>|*z*|)
(Intercept)	82.213	36.13	2.276	**0.0229**
Original first-order interquartile range	9.148	10.075	0.908	0.3639
Wavelet-HHH first-order skewness	-273.718	122.651	-2.232	**0.0256**

H: high-pass filter. Bold values represent that the results have statistical significance.

## Data Availability

All the raw data could be accessed by contacting the corresponding author upon need.
